The article "Body Weight Is a Valid Predictor of the Long-Term Prognosis of Cervical Cancer" was published in 2022. Journal: Comput Math Methods Med.

# Body Weight Is a Valid Predictor of the Long-Term Prognosis of Cervical Cancer

**DOI:** 10.1155/2022/5613350

**Published:** 2022-06-08

**Authors:** Li Lu, Shuqi Ji, Jing Jiang, Yu Yan

**Affiliations:** Department of Obstetrics and Gynecology, 2nd Affiliated Hospital of Harbin Medical University, China

## Abstract

**Objective:**

To identify and validate effective clinical predictors for the long-term prognosis of patients with cervical cancer.

**Methods:**

Cervical cancer patients were retrieved from the TCGA database, and patients' clinical data were collected and analyzed for the predictive value of long-term prognosis. In the other branch of the study, patients with cervical cancer and admitted to our hospital between January 1, 2016, and December 31, 2016, were retrieved and followed up for prognosis analysis.

**Results:**

In the database patient cohort of our study, 607 cases with cervical cancer were analyzed. Aneuploidy score (*p* = 0.012), Buffa hypoxia score (*p* = 0.013), histologic grade (*p* = 0.01), fraction genome altered >0.4 (*p* < 0.001), weight > 60 kg (*p* < 0.001), height > 160 cm (*p* = 0.047), BMI <18.5 (*p* = 0.023), Winter hypoxia score (*p* = 0.002), and adjuvant postoperative radiotherapy were good predictors for disease-free survival (DFS), while aneuploidy score (*p* = 0.001), MSI sensor score > 0.5 (*p* = 0.035), person neoplasm status (*p* < 0.001), race (*p* = 0.006), Ragnum hypoxia score (*p* = 0.012), weight (*p* < 0.001), height (*p* < 0.001), and BMI < 18.5 (*p* = 0.04) were good predictors for overall survival (OS). In the admitted patient cohort, age over 60 years old at the time of diagnosis was the only clinical factor influencing the long-term DFS (*p* = 0.004). TNM stage above III (*p* = 0.004), body weight > 70 kg (*p* < 0.001), and complicated with other cancer (*p* < 0.001) were clinical factor influencing the long-term OS.

**Conclusions:**

Clinical factors, especially common to both cohorts, could be used to show the long-term prognosis of cervical cancer.

## 1. Introduction

The American Cancer Society predicts that in the year of 2022, there will be about 14,100 women who will be new cases of invasive cervical cancer, and about 4,280 women who will die from cervical cancer [1]. All over the world, women diagnosed with or died from cervical cancer in 2020 were estimated to be 604,127 or 341,831, respectively [2]. Thanks to the screening methods of Pap smear test and the recent detection of human papilloma virus (HPV) subtypes, both the incidence and the deaths caused by cervical cancer have been decreasing over the past 40 years in the United States [3].

Cervical cancer may present with different symptoms and signs at different clinical stages, from none at early stages (about 44% of cervical cancer are diagnosed at this stage) to vaginal bleeding after intercourse between periods or after menopause, bloody vaginal discharge, or pain during intercourse at more advanced stages.

Serum or cancer tissue biomarkers for the prediction of prognosis of cervical cancer have been reported [4, 5]. The 5-year survival rate for overall cervical cancer is 66%, which is affected by race, ethnicity, age, and stage [2]. But the efficacy of those clinical factors in the prediction of prognosis of cervical cancer might be different due to the differences in race, genetic factors, living habits, and economic conditions across the world.

In this study, we investigated the efficacy of clinical factors in the prediction of the prognosis of patients with cervical cancer. We first analyzed data collected from a public database and then analyzed and validated the findings in patients admitted to our hospital. We found that aneuploidy score, Buffa hypoxia score, histologic grades, fraction genome altered, weight, height, BMI, Winter hypoxia score, adjuvant postoperative radiotherapy, MSI sensor score, person neoplasm status, race, Ragnum hypoxia score were important clinical predictors for the 5-year prognosis of cervical cancer in patients from database, while age, TNM stages, and body weight, diagnosed with other cancer, were important clinical predictors for the 5-year prognosis of cervical cancer in patients admitted to our hospital.

## 2. Materials and Methods

### 2.1. Patients

We searched the TCGA database (https://cancergenome.nih.gov) and identified the cervical squamous cell carcinoma dataset (*n* = 297) and the cervical squamous cell carcinoma and endocervical adenocarcinoma dataset (*n* = 310). All cases with available information were included for analysis. Clinical data of patients diagnosed with primary cervical cancer and admitted to our hospital between January 1, 2016, and December 31, 2016, were retrieved for analysis. Patients were followed up for prognosis information. This study was approved by the ethical committee of our hospital. Informed consents were obtained during follow up.

### 2.2. Data Extraction

Clinical characteristics, including age, disease-free survival (DFS), overall survival (OS), race, clinical stages, histologic grades, mutation count, weight, height, BMI, and postoperative radiotherapy, were extracted from the databases as well as patient records from our hospital.

### 2.3. Statistical Analyses

The measurement data were expressed as mean ± standard deviation (SD). The Kaplan-Meier survival curve was employed to show the correlations between clinical characteristics and long-term prognosis, including DFS and OS. The receiver operating characteristic (ROC) curve was employed to show the effectiveness of clinical characteristics to predict 5-year survival. Statistical analyses were performed using SPSS 24.0 (SPSS Inc., Chicago, USA). A two-tailed *p* value of less than 0.05 was determined as statistically significant.

## 3. Results

### 3.1. Clinical Characteristics

There were 607 patients collected from the two TCGA database (Table 1). The mean age at diagnosis was 48.2 ± 13.8 years old, with a mean DFS of 34.2 ± 32.7 months, a mean OS of 33.3 ± 37.0 months, and a mean body weight of 73.1 ± 21.5 kg. Height, weight, TNM stage, histologic stage, fraction genome altered, race, lymphovascular invasion indicator, neoplasm status, and mutation count were further analyzed (Table 1). On the other hand, ninety-four qualified patients were retrieved from the medical record at our hospital, and the complete data collected from 61 cases during our follow-up contact were collected and analyzed. The mean age of followed-up patients were 47.6 ± 9.1 years old, with a mean DFS of 59.2 ± 4.8 months, a mean OS of 58.0 ± 7.0 months, and a mean body weight of 61.0 ± 7.3 kg.

### 3.2. Determination of Predictive Factors for DFS in Database Patients

Aneuploidy score (*p* = 0.012), Buffa hypoxia score (*p* = 0.013), histologic grade (*p* = 0.01), fraction genome altered >0.4 (*p* < 0.001), weight > 60 kg (*p* < 0.001), height > 160 cm (*p* = 0.047), BMI <18.5 (*p* = 0.023), Winter hypoxia score (*p* = 0.002), and adjuvant postoperative radiotherapy (*p* = 0.017) were all significantly correlated with disease-free survival, whereas age at diagnosis, lymph node stage, tumor stage, squamous cancer, person neoplasm status, race, Ragnum hypoxia score, corpus uteri involvement, total number of pregnancies, cigarette smoking, and hysterectomy type were not (all *p* > 0.05, Table 2). Kaplan-Meier survival curves, as well as the corresponding ROC curves were shown in Figure 1. When judged by the area under the curve, weight < 60 kg showed the best value (area = 0.837) in prediction of long-term DFS.

### 3.3. Determination of Predictive Factors for OS from Database Patients

Aneuploidy score (*p* = 0.001), MSI sensor score > 0.5 (*p* = 0.035), person neoplasm status (*p* < 0.001), race (*p* = 0.006), Ragnum hypoxia score (*p* = 0.012), weight (*p* < 0.001), height (*p* < 0.001), and BMI< 18.5 (*p* = 0.04) were significantly associated with OS (Table 3). On the other hand, age at diagnosis, clinical stages, histologic grade, fraction genome altered, MSI MANTIS score, mutation count, corpus uteri involvement, Winter hypoxia score, adjuvant postoperative radiotherapy, total number pregnancies, cigarette smoking, and hysterectomy type were not correlated with OS (all *p* > 0.05, Table 3). Kaplan-Meier survival curves and ROC curves of corresponding factors were shown in Figure 2. Based on the area under the curve, Ragnum hypoxia score and MSI sensor score > 0.5 both showed the best value (area = 0.594) in prediction of long-term OS.

### 3.4. Predictive Factors for Admitted Patients

Age over 60 years old at the time of diagnosis was the only clinical factor influencing the long-term DFS (*p* = 0.004). TNM stage above III (*p* = 0.004), body weight > 70 kg (*p* < 0.001), and complicated with other cancer (*p* < 0.001) were clinical factors influencing the long-term OS (Table 4). In the corresponding ROC curves, age over 60 years had an area under the curve of 0.942 for the prediction of long-term DFS, whereas weight > 70 kg had an area under the curve of 0.722 for the prediction of long-term OS (Figure 3).

## 4. Discussion

In this study, due to the limited availability of many clinical exams, a lot of clinical factors determined to be predictors of the prognosis of cervical cancer in the database patient cohort could not be validated in our admitted patient cohort. Among clinical factors available in both database and admitted patients, there were still quite a lot of differences. Histologic grades, body weight, and adjuvant postoperative radiotherapy were predictive factors for database patients' DFS, whereas age > 60 years was the only predictive factors for admitted patients' DFS. On the other hand, body weight was the only predictive factors for database patients' OS, whereas TNM stage, body weight, and complicated with other cancer were the predictive factors for admitted patients' OS.

The finding of body weight as a predictor for the prognosis of cervical cancer patients coincided with a recent study, where patients received concurrent chemoradiotherapy [6]. However, only 159/547 (29%) of database patients and 34/61 (56%) of admitted patients in our study received adjuvant postoperative radiotherapy, suggesting the efficacy of weight or BMI as predictive factors for the prognosis of cervical cancer does not rely on chemoradiotherapy, but was really related to cervical cancer itself.

In the database cohort, 163/302 (54%) patients were diagnosed at clinical stage I, 70/302 (23%) at clinical stage II, 47/302 (16%) at clinical stage III, and 22/302 (7%) at clinical stage IV, whereas in the admitted cohort, 17/61 (28%) patients were diagnosed at clinical stage I, 34/61 (56%) patients were diagnosed at clinical stage II, 5/61 (8%) patients were diagnosed at clinical stage III, and 5/61 (8%) patients were diagnosed at clinical stage IV. The later stage at diagnosis in our admitted patients cohort suggests a late detection, which might reflects a lower rate of annual Pap smear and/or HPV screening, as well as the lower availability of HPV vaccination in China. Also, the finding that clinical stage showed a good predictive value as a predictive factor for the OS of cervical cancer in the admitted cohort, but not in the database cohort, might be due to the relatively higher percent (more weight) of clinical stage II patients.

The evolving development in big data techniques makes data mining from published database a feasible and affordable way for clinical studies [7, 8], although the inconsistency in study design and retrospectively collected data make a lot of parameters incomparable between different studies [9]. Ideally, comprehensive parameters in the field of psychology and social-economy need to be obtained for a better understanding of factors influencing the prognosis of cervical cancer. Interesting topics might include income, nutrient conditions, anxiety, depression [10], living habits, etc. In our admitted cohort, we included the parameter of “self-living,” which, although did not show significant contribution to the long-term prognosis, was still near to statistical borderline (*p* = 0.07) and might be a promising factor if we include more cases in the future. Other clinical conditions, such as histories of labor induction [11], treatment of preterm labor [12], fulminant hepatitis [13–16], role of RNA interference [17], and HPV [18], might also contribute to the prognosis of cervical cancer.

To sum up, we found clinical factors, especially body weight, histologic grades, age, TNM stages, complicated with other cancers, and adjuvant postoperative radiotherapy, can be valid long-term predictors of prognosis of cervical cancer. A uniformed reporting system is needed for the benefit of future updates and analyses.

## Figures and Tables

**Figure 1:** Kaplan-Meier survival curve and ROC curve of predictive value of clinical factors for DFS in database patients.

**Figure 2:** Kaplan-Meier survival curve and ROC curve of predictive value of clinical factors for OS in database patients.

**Figure 3:** Kaplan-Meier survival curve and ROC curve of predictive factors for DFS and OS in admitted patients.

**Table 1:** Characteristics of analyzed patients from database (n = 607).

Variable	Mean ± SD or subgroup	*n*
Age at diagnosis (years)	48.2 ± 13.8	606
Weight (kg)	73.1 ± 21.5	548
Height (cm)	161.0 ± 7.3	265
DFS (months)	34.2 ± 32.7	242
OS (months)	33.3 ± 37.0	606
Clinical stage	IA	8
	IB	155
	IIA	26
	IIB	44
	IIIA	4
	IIIB	43
	IV	22
Histologic grade	I	36
	II	267
	III	237
	IV	2
	X	17
Race	White	415
	Black	59
	Asian	40
	American Indian	16
	Pacific islander	4
Fraction genome altered	0.27 ± 0.18	293
Lymphovascular invasion indicator	Yes	82
	No	72
Neoplasm status	Tumor free	376
	With tumor	146
Mutation count	180.3 ± 571.2	475

**Table 2:** Clinical factors for the prognosis of DFS of patients from database.

Clinical factors	*p* value (DFS)	*n*
Age at diagnosis (years)	0.773	242
Lymph node stage	0.959	206
Tumor stage	0.856	202
Squamous cancer	0.245	242
Aneuploidy score	0.012	170
Buffa hypoxia score	0.013	170
Histologic grade groups	0.01	239
Fraction genome altered (>0.4)	<0.001	242
Person neoplasm status	0.056	211
Race	0.322	211
Ragnum hypoxia score	0.3	123
Weight (<60 kg)	<0.001	222
Patient height (<160 cm)	0.047	107
BMI< 18.5	0.023	93
Corpus uteri involvement	0.641	56
Winter hypoxia score	0.002	118
Adjuvant postoperative radiotherapy	0.017	69
Total number pregnancies	0.829	103
Cigarette smoking pack year	0.055	35
Hysterectomy type	0.213	75

**Table 3:** Clinical factors for the prognosis of OS of patients from database.

Clinical factors	*p* value (OS)	*n*
Age at diagnosis (overall)	0.425	602
Lymph node stage	0.349	512
Tumor stage	0.998	484
Cancer type	0.849	604
Squamous	0.257	604
Aneuploidy score	0.001	293
Histologic grade	0.168	589
Fraction genome altered	>0.05	297
MSIMANTIS score	>0.05	297
MSI sensor score	>0.05	297
MSI sensor score (>0.1)	<0.001	297
MSI sensor score (>0.2)	<0.001	297
MSI sensor score (>0.5)	0.035	297
MSI sensor score (>1)	0.572	297
Mutation count	>0.05	533
Person neoplasm status	<0.001	522
Race	0.006	534
Ragnum hypoxia score	0.012	293
Patient weight (overall)	<0.001	547
Patient height (overall)	<0.001	265
Patient height (< 170 cm)	0.01	265
BMI (overall)	0.032	218
BMI (<18.5)	0.004	218
Corpus uteri involvement	0.289	118
Winter hypoxia score	>0.05	293
Adjuvant postoperative radiotherapy	0.941	159
Total number pregnancies	0.174	269
Cigarette smoking pack year	>0.05	95
Hysterectomy type	0.39	170

**Table 4:** Predictive factors for survival of admitted patients.

Variable	Cutoff	*p* value of DFS	*p* value of OS
Age at diagnosis (years)	Overall	0.38	0.25
	>30	0.85	0.65
	>40	0.73	0.41
	>50	0.16	0.46
	>60	0.004	0.1
TNM stage	Overall	0.87	0.004
	II	0.53	0.49
	III	0.71	0.004
	IV	0.85	<0.001
Histologic grade	Overall	0.28	0.17
	II	0.57	0.61
	III	0.11	0.13
Radiation and/or chemotherapy	Yes	0.68	0.53
Body weight (kg)	Overall	0.98	0.005
	>50	0.73	0.41
	>60	0.31	0.36
	>70	0.76	<0.001
Smoke	Yes	0.81	0.57
Longest dimension of lesion (cm)	Overall	1.00	0.65
	>1	0.70	0.88
	>2	0.34	0.12
	>3	0.18	0.98
	>4	0.72	0.39
Other cancer		NA	<0.001
Self-living	Yes	0.89	0.07

## Data Availability

The datasets used in this study are available from the corresponding author on reasonable request.
